RETRACTED

# Extracting Behavior Identification Features for Monitoring and Managing Speech-Dependent Smart Mental Illness Healthcare Systems

**DOI:** 10.1155/2022/8579640

**Published:** 2022-05-06

**Authors:** Alka Londhe, P. V. R. D. Prasada Rao, Shrikant Upadhyay, Rituraj Jain

**Affiliations:** ^1^Department of Computer Science and Engineering, Koneru Lakshmaiah Education Foundation, Vaddeswaram, AP, India; ^2^Department of Electronics & Communication Engineering, Cambridge Institute of Technology, Ranchi, Jharkhand, India; ^3^Department of Electrical and Computer Engineering, Wollega University, Nekemte, Ethiopia

## Abstract

Speech is one of the major communication tools to share information among people. This exchange method has a complicated construction consisting of not the best imparting of voice but additionally consisting of the transmission of many-speaker unique information. The most important aim of this research is to extract individual features through the speech-dependent health monitoring and management system; through this system, the speech data can be collected from a remote location and can be accessed. The experimental analysis shows that the proposed model has a good efficiency. Consequently, in the last 5 years, many researchers from this domain come in front to explore various aspects of speech which includes speech analysis using mechanical signs, human system interaction, speaker, and speech identification. Speech is a biometric that combines physiological and behavioural characteristics. Especially beneficial for remote attack transactions over telecommunication networks, the medical information of each person is quite a challenge, e.g., like COVID-19 where the medical team has to identify each person in a particular region that how many people got affected by some disease and took a quick measure to get protected from such diseases and what are the safety measure required. Presently, this task is the most challenging one for researchers. Therefore, speech-based mechanisms might be useful for tracking his/her voice quality or throat getting affected. By collecting the database of people matched and comparing with his/her original database, it can be identified in such scenarios. This provides the better management system without touching and maintains a safe distance data that can be gathered and processed for further medical treatment. Many research studies have been done but speech-dependent approach is quite less and it requires more work to provide such a smart system in society, and it may be possible to reduce the chances to come into contact with viral effected people in the future and protect society for the same.

## 1. Introduction

### 1.1. Background and Principle of Speaker Recognition

In this respect, speech supplies naturally and handily the shape of an entry that conveys a remarkable amount of speaker supporting information, and it is cheap to analyze and collect.

RETRACTED

Voice is an occurrence that extremely relies on the speaker who generates it. Various physical outlooks of speech such as tone, timber, or intensity vary plenty from a speaker to another. The similar happens with supplementary linguistic aspects such as the individual intonation and expressions a speaker normally uses or a range of vocabulary [1, 2]. All these belongings make voice a very strong biometric essential to be implemented in security structure since the physical attribute of speech is easy to calculate and compare in comparison with other biometric essentials and other medical issue analysis. The speed-dependent technology leads to better control without touching and maintaining a safe distance for information gathering for subsequent medical treatment in the healthcare system. It also protects society by decreasing the possibility of coming into touch with a virally affected individual in the future. In inclusion, the speech wave is quite well known and has been greatly studied for many years, so many powerful algorithms can be found to deal with this kind of signal [3].

Textual content-dependent project entails a form of predicated or triggered passwords as a way to achieve the required textual content. It could be used for packages consisting of voice method signature or password confirmation. In aforesaid programs, there is a need to alternate the key or password; often it is smart to make completed without difficulty through converting the predicated text. In text-based speaker verification, at some point of the enrolment segment, a limited number of utterances of constant textual content are amassed [4]. The proposed model is more secure than the previously implemented models. This management approach, which uses speech samples, reduces the number of persons in contact, breaks the mass into pieces, and provides a better option for dealing with such a situation. Consequently, approaches primarily based on template matching are used for sample contrast rather than procedures primarily established on facts having feigned neural grids, which requires a massive quantity of learned records. Studies in the processing of speech and verbal exchange, as the maximum element, influenced by means of humans, wish to construct mechanicals prototypes to imitate human lexical conveying [5–7]. Speech processing research interest in these days is performed properly beyond the conception of copying human spoken equipment. Biomedical gains attention in different applications such as real voice analysis, operation work functioning, and viral infected throat identification [8, 9].

RETRACTED

Addresser popularity is a system of unconsciously spotting who is expressing through the use of speaker unique statistics blanketed in speech gestures to confirm the recognition being stated via human being retrieving systems; that is, it permits to get admission to manage of diverse offerings by way of voice. Speaker identification is matched up to the anatomical and behavioural properties of the speaking manufacturing machine of a separate speaker. These properties deduce from each insubstantial pouch (vocal span properties) and prosodic capabilities (input supply traits) of articulation. The bulk usually worn quick-time period ghastly estimations cestrum measures and their throwback measures. Therefore, for the throwback measures, usually the primary and 2nd-order measures, this is subordinate to the pulse functions of cestrum measures, which are retrieved at each body cycle, to symbolize the ghastly energetic. Those throwback measures are also known as delta-cestrum and delta2cepstralmeasures [10].

The present article has been planned into various sections. Section 1 deals with introducing the concept and principle of speaker recognition. Section 1.1 puts light on the discussion of related research work. Section 2 illustrates the automatic addresser identification. Section 3 describes the recognition, spotting, and validation. Section 4 describes the preparation of database. The proposed model and results are described in Section 5, and finally Section 6 portrays the conclusion and possible future works based on the proposed framework.

### 1.2. Literature Review

Speaker verification stands on the belief that there is always some quality in every person's speech and that it can be used to verify his/her identity. The quality features in speakers' voices are used both to train a user model and to make up a reference identity for the claimed cause to be used for verification against the user's model. Feature extraction by Schmid and Gisht, 1994, suggested that the first stage of taking out information from a speech signal is known as feature extraction [10]. Both have also discussed that speech information is essential for different speech processing tasks such as speaker verification is taken as a short spectrum; as per the same author, spectral information is captured during a period of about 20 ms [11].

On the other side, Furui, 1997, discussed that an effective method to differentiate between users in a system is fundamental frequencies and different measurements of signals similar to long-term spectrum and short-term spectrum and in all powers. Gold and Morgan, 2000, discussed that text-independent and text-dependent focus on a client's input (voice) is naturally relied on process for verification [12]. For speech recognition, the correct action of speaking in terms of features is contingent on the classification technique being used. Anyhow, in some system types, Morgan and Gold, 2000, whether the verification is text-dependent, text-independent of some different group, the estimated claimant of a user model always needs the score calculation that informs the system about the distinguishable/indistinguishable vocal sounds, or statements of the claimant are matched to the model [13]. Clearly, a comparison is performed between the feature extracted and the features that the speaker model for the claimant is standing on the comparison of their spectra or both can be evaluated using statistical measures, on the basis of certainty/uncertainty between the model and the claimant's voice [14]. Morgan and Gold, 2000, also investigated that acoustic aspect degree is not frequently used as the statistical degree. Doddington, 1998, Furui, 1997, and Schmidt and Gish, 1994, discussed the environmental effect on the speech signal coming from different sources, for example, acoustic noise Doddington, 1998, and different transmission and recording environments for speech Doddington 1998, Furui, 1999 and environmental sound or other interfering voices Schmidt and Gish, 1994 [15].

RETRACTED

A text-dependent system has no advance knowledge; whatever it may be, the claimed will throw during the session (Den Os and Boves & Doddington, 1998); therefore, it will accept or reject his/her request on the characteristics of his/her voice. This is because of reality that the system does not use vocabulary understanding, and achievements become poor compared with the text-dependent system [16].

Blombug in 2002 has underlined the major structure classes from the number of text-reliant to the number of text-self-reliant.

1. Text-reliant has a prearranged (fixed) key
2. Text-reliant defined key for every user
3. One's voice dependent
4. Action dependent, i.e., certain phonemes
5. System chooses the text (text-independent)

Fletcher, 1938, located the idea of a critical band that the edge of listening to change into detected for a sinusoid wave as a purpose of transmission capability of a band-allowed noise and counselled that the human auditory machine behave. Although it consisted of a group of round-skip filters having overlie skip band which introduces the period essential bandwidth [17].

### 1.3. Humans Associated with Speaker Recognition

Human beings can reliably discover acquainted voices and approximately two to three seconds are sufficient to perceive a voice despite the fact that altogether showing decrease in unusual inputs (voice). Surprisingly, if length of the statement becomes expanded, however, performed in reverse (which disturbs the schedule and utterance prompts), the precision reduces extensively. Extensively various overall performances in the historical past challenge recommended, that prompts to input voice popularity range from voice to voice, and that voice styles might also include a fixed set of auditory prompts from where audiences pick out a subgroup to apply in figuring out separate inputs (voices) [18]. Reputation frequently drops drastically while addressers strive to discriminate their inputs (voices). This pondered in appliances, in which precision is reduced while imitating behaves as hoaxers. Speaker reputation is a single location for synthetic observation where gadget overall execution can excel human overall execution, with the usage of quick take a look at observations and N-quantity of audio system, the system precision regularly excels that of humans. This is in particular for a strange audio system in which the education time for human beings to adopt or examine an updated input (voice) is generally too lengthy as contrast to that for systems (machines). Persons overall production in unfavourable situations changed into additionally judged wherein it changed into stating definitely that human listeners adopt the use of numerous cues to affirm the audio system in the presence of acoustic mismatch [19, 20].

RETRACTED

### 1.4. Recognition Process

Speaker reputation of the system (machine) requires 3 ranges; they are (1) removal of functions to denote the addresser details near the articulation signal; (2) designing of addresser qualities; and (3) choice common sense put into effect for identity or validation challenge. The issues related to each of these stages are discussed as follows.

The primary project in an addresser popularity machine or model is to remove attributes capable of indicating the addresser facts existing in the articulation sign. It is regarded that human beings use high-stage capabilities along with the fashion of speech, speech, dialect, and verbal mannerisms (as an example, a particular kind of amusing or use of unique idioms and words) to understand speakers. Intuitively, it is far clear that those functions constitute crucial speaker statistics. Issue arises because of obstacles of the present characteristic extraction strategies. Current speaker recognition systems comply with segmental features inclusive of a pattern for the vocal tracts to symbolize speaker precise information[21]. These capabilities show sizeable versions across speakers; however, they also display sizable versions now and then for an unmarried speaker. In addition to this, the traits of the recording device and transmission channel are also meditated in these capabilities. As soon as a right set of function vectors is acquired, then within the next section the assignment of addresser identification is to generate a version (archetype) for each addresser [22]. The growth of addresser modelling is referred to as the training section. The schematic diagram of the learning phase is shown in Figure 1.

RETRACTED

Characteristic polar coordinates showing the voice quality of the addresser are taken out and worn for constructing the testimonial fashions. Performance of a speaker popularity machine depends in general on the effectiveness of the model in taking pictures and speaker-specific records, and therefore this phase performs a chief function in figuring out the overall performance of a speaker reputation device [23]. The final level inside the improvement of a speaker reputation machine is the decision common sense degree, where a choice to either take delivery of or to refuse the affirm of an addresser is received based totally on the end answer of the complement strategies used. The illustration of choice, good judgment, and testing segment method is shown in Figure 2.

## 2. Automatic Addresser Identification

Addresser reputation generally consists of various extraordinary approaches of discerning humans depending totally on their voices. The main classes are addresser recognition and addresser verification [24].

In addresser recognition, a speech observation from the hidden addresser is judged and compared with the prototypes of all acknowledged speakers. The hidden addresser is recognized as the speaker whose prototype best suits the input observation.  Figure 3 suggests the plain structure of the addresser identity machine [25].

Addresser identity can be a confined set identity or unlock set identity. In a lock set spotting, it is far considered that the check utterance belongs to one in all N enrolled speakers (N decisions). In the case of open set identity, there may be an extra decision to be made to decide whether to take a look at the utterance changed into uttered by way of one of the N enrolled speakers or now not; this is, there are *N* + 1 selection degrees [24, 25]. The addresser's speech character is represented by characteristic polar coordinates, which are removed and used while generating the testimony. The success of the algorithms in collecting the speaker-specific defines the overall efficiency of a speaker popularity machine; hence, this stage is important in determining the actual quality of a speaker popularity machine.

RETRACTED

Addresser verification objective is to just allow or disallow the affirm of the addresser based totally on the samples of his speech. If the healthy check and reference are above a positive entrance, declare is regular. A high entrance makes it hard for pretenders to be normal by using the machine but with the danger of disallowing the real individual. Conversely, a low entrance ensures that the real person is widely wide-spread continuously, however, with the chance of accepting impostors [26].  Figure 4 suggests the simple structure of a speaker verification machine.

### 2.1. Approaches Adopted for Speaker Recognition

Early research on text-independent speaker reputation is used averaging of function vectors to create a reference template. In the correlation matrices derived from the spectra of an incredibly long length of speech, alerts are used to specify speaker differences. In this research, speech is very useful for remote attack transactions across telephone networks, medical data, and healthcare systems. As a result, a speech-based technique might be effective in detecting changes in voice quality or throat irritation. Persons can be identified in such a setting by gathering a database of people who matches the original database. This allows for a better management system in healthcare. Such techniques will not correctly represent the distribution of characteristic vectors which are modelled by means of parametric or nonparametric methods. Fashions which expect a chance density feature are termed parametric. In nonparametric modelling, minimal or no assumptions are made regarding the chance distribution of function vectors. In this segment, we in brief evaluate the exclusive version like Gaussian combination version (GMM), Hidden Markov model (HMM), Vector Quantization (VQ), and neuronal community primarily based procedures for speaker reputation. GMM and HMM are parametric fashions [27–29]. VQ and neural network models are dealt as nonparametric models. The Hidden Markov model (HMM) has been the foundation of a number of effective acoustic modelling approaches in speech recognition systems. The model's analysis skill in phenomena, as well as its effectiveness in real voice recognition systems, is the prime cause for its achievement.

Addresser authentication is an unlatched problem. Addresser authentication structures can be additions categorized as textual content-based and textual content-impartial process. Inside the text-attached addresser recognition device, the word to be spoken is fixed. In a self-reliant text addresser recognition device, there may be no restrictions on the text to be spoken. Usually, a textual content-based speaker verification machine performs better than a textual content-impartial speaker verification system due to the high degree of control exercised over the speech sign conditions [30]. The text-dependent and text-independent can be described with the help of an example to make it clearer as shown in Table 1. In the initial stage, the agents are verified by some mean of password, and in the second step, the agent will be verified by using the voice giving some numeric value to the system. The most important comparison among HMM, VQ, and neuronal communities is the Hidden Markov model (HMM) dealing with limited factions, while vector quantization and neuronal community are nonparametric models.

RETRACTED

### 2.2. Importance of Feature Extraction

Speech signal carries the following information:

- The intended message
- Language spoken
- The speaker's Identity
- The emotional and physical state of the speaker

Feature removal is the approximation of variables called feature vectors, which loyally describe the pattern (speech pattern) and the problem under deliberation (speaker recognition). The main purpose of the feature removal phase in speaker identity is to withdraw the speaker precise satisfactory [31].

Voices of any two persons vary due to the dissimilarity in the diameter of the spoken space, dissimilarity in the size of the spoken strings, and the fashion in which they are used to generate speech. The short-duration spectrum is chiefly identified by the vocal stretch. Parameters of the characteristics interconnected with the spectrum are acquired from a tiny segment (typically10–30 msec) of the speech signal, and that is why they are called segmental characteristics. The dissimilarity in the speaking way is due to the way in which the speaker has learned to apply his/her speech production mechanism [32–34]. The temporal dissimilarities of speech traits of various individuals are indicated by these differences. These characteristics are generally eliminated from a comparatively long segment (usually 100–300 msec) of the speech signal, and thus these characteristics are called suprasegmental characteristics. It is visible that all characteristics taken out should be chosen for speaker acceptance. Therefore, as the feature vector size increases, the computation and storage necessity also increase. For that reason, there is a demand for quality elections. The intention of quality choice is to take a look at the changes in a comparatively low dimensionally quality space that holds the data suitable for the software. At the similar duration, it should also be feasible to accomplish meaningful differentiation using simple actions.

RETRACTED

## 3. Recognition, Spotting, and Validation

Addresser reputation may be divided into subtasks, i.e., addresser spotting and validation. Addresser identity indicates identity for the addressers, wherein addresser validation is a system of accepting or reusing as the recognizer of declared users. Morgan in 2000, Gold, 1997, and Doddington, 1998, used terms when talking about speaker perception and speaker spotting.

Speaker verification is basically a category with two sections; the training session: it is when a model of the user's voice is built up and the real verification is done. The system is thus trained first for a new user's voice that can be performed in many sections, which mean that a spectral analysis is done from which features are extracted to generate a speaker model [35].

Secondly, the user's voice can be verified by comparing the claim's voice with the trained database of user models. On a comparison basis, the system will decide whether the claim's identity is the one modelled by the training material or not. Speaker verification stands on the belief that there is always some quality in every person's speech and that it can be used to verify his/her identity. The quality features in speakers' voices are used both to train a user model and to make up a reference identity for the claimed cause to be used for verification against the user's model [36].

Murray et al., suggested that the first stage of taking out information from speech signal is known as feature extraction. Both have also discussed that speech information is essential for different speech processing tasks [37] like speaker verification is taken as a short spectrum; as per the same author, spectral information is captured during a period of about 20 ms.

On the other side, Furui, 1997, discussed that an effective method to differentiate between users in a system is fundamental frequencies and different measurements of signals similar to long-term spectrum and short-term spectra and in all powers.

Gold and Morgan, 2000, discussed that text-independent and text-dependent focus on a person's voice is naturally relying on the process of verification. For speech recognition, the correct action of speaking in terms of features is contingent on the classification techniques being used [38].

Doddington, 1998, Furui, 1997, and Schmidt and Gish, 1994, discussed the environmental effect on the speech signal coming from different sources, for example, acoustic noise by Doddington, 1998, and different transmission and recording environments for speech by Doddington 1998, Furui, 1999, and environmental sound or other interfering voices by Schmidt and Gish, 1994.

RETRACTED

Doddington, 1998, also stated that differences in the speaker's voice or between different speakers affect the quality of the speaker verification system and suggested that some of the factors that influence and highlight that one justification for speaker voice changes is that the use of speech is a consequence of a person [39]:

1. Psychical health and physical condition
2. Age factor (human's voice changing as he/she is getting older)
3. Speaking rate and level of speech effort
4. Intelligence and educational level
5. Verification system is experienced

### 3.1. Model for Speech Recognition

The GMM became first added through Rose and Reynold, 1995, and was an especially used speaker model as it has the potential to model random desire, fashioning possibility density capabilities (pdfs), with the usage of superposition of multivibrate Gaussian. For the diagonal covariance matrix, this is even genuine when the loss in expressible induced by using the Gaussians being restrained to a round area which may be struggling with the usage of more Gaussians. Using diagonal covariance will help to enhance reputation performance, and much less parameters of the model may be predicted greater comfortably from the limited education facts. The main purpose for deciding on such a model system is that everyone aggregate fashions a hid massive speech sound class [16]. GMM consists of a combination of *M* Gaussians, in which *M* absolutely relies nonlinearly on the context and length of the training records supplied through the user [40]. The proposed method is based on speech-dependent health monitoring and management system. In this system, the speech signal may be used to identify a variety of symptoms, such as throat infection, speech pattern alignment, or any voice-related issues.

The classical value of “M” is 32 for characteristics attribute dimensions in the span of 12 to 26. D-dimension is employed for each mixture with mean vector □(⟶┬*μ*) and diagonal covariance vector □(⟶┬*σ*^2), measured by the agent “w” so that the total mass is 1 and modelling shape is scattering. The log-likelihood l_GMM for D-dimensional feature vector *X*={□(⟶┬*y*_*t*)*|*1 ≤ *t* ≤ *T*∧□(⟶┬*y*_*t*) ∈ *S*  *D*} given by the probability *P*(*X|λGMM*) is represented by its parameter. Gaussian chance distribution and capabilities belonging to the clusters may be satisfactory and acceptable through their opportunity values. The best problem includes green category of feature vectors [41, 42].  Figure 5 shows the Gaussian Mixture Model with its feature space and corresponding 2-dimension.

GMM used for speaker identification is influenced by two facts as follows Gaussian individual classes are explained to represent the acoustic class, and its set vocal tract information represents the acoustic classes.

RETRACTED

GMM density gives a uniform approximation to the distribution of feature vectors in a multidimensional region.

### 3.2. Functioning of Health Unit

Health centre generates an authenticated report on the basis of his/her voice quality or speech analysis and generated throat quality analysis parameters using a feature extraction method which may or may not be the same as per the original speech quality as saved in database.

Monitoring will be done on the basis of speech data collected per data, and its testing will be done *n* number of times using training, training, and sampling techniques which may hardly take a few milliseconds. Smart management is the need of an hour where the situation changes suddenly and monitoring is required at every point of time. Pandemic situations may occur in the future, and such challenges require regular monitoring and real-time management systems to deal with such scenarios. COVID-19 [43] affected the entire nation, and India is the only country where the recovery rate is quite high compared with other developed nations in spite of low medical facilities, and everybody is not capable to have a medical test in terms of blood samples and get the result fast. However, many people face difficulties in rural areas where the situation is the worst, and the testing rate is very slow and needs more attention. In such condition, voice can be used to collect the sample of each person by taking the sample just by making a call and matching process by extracting the feature, and sampling may be useful. The only thing required is to make a database of villagers in terms of speech and store in the cloud and can be accessed anywhere and verification can be done anytime. The data collection centre can gather the information in terms of speech, and that sample will be analyzed using its original sample and trained by the system and matched with the saved database sample by extracting its original frequency spectrum variation, and it will be verified, and finally the control room of the hospital will generate a report by analyzing various parameters of voice and sent to the person whose voice really gets disturbed and might not be affected by some viral disease or voice disorder as shown in Figure 6.

## 4. Preparation of Database

The bottom has been organized for fifty audio systems collecting the samples (spoken) of males and females of various group institutions, with the usage of gold wave 5.5 and cool tool program using microphones. The directory collected outlying Hindi numbers along with 0, 1, 2, 3, 4, 5, 6, 7, 8, and 9. Every addressers speak 0–9 digits (in Hindi), each number for 10 instances, then changed into a note in a noise-unfastened condition, and kept as a wave sound file (.wav) recording the desired folder.  Table 2 shows the full database of 50 different speaker users including both males and females of different groups. The parameters of data/sample collection are shown in Table 3.

RETRACTED

### 4.1. Procedure for Data Collection

The spoken of 50 distinctive audio systems has been put down the usage of taxon speakers. Every spectrum of Hindi text from 0 (SHUNYA) to 9 (NAU) was spoken 10 times, and every text has been put down inside the shape of the scale by reducing each scale (frame), and via choosing “store alternative” from the record menu, each scale is stored using.wav file in a suitable folder. The spectrum of Hindi digits is recorded using cooling software which reflects different energies.

Steps involved are as follows:

1. First, choose the application type; it will give the blank space in Graphical User Interface type (GUI).
2. Go to the file menu and select new.
3. This will give the option to choose sampling rate, channels, and resolution.
4. Then, press OK by selecting the proper sampling rate, channel, and resolution; it will give a blank space.
5. Now, go the record option indicated in the left bottom corner and press the record button to record the Hindi spoken digits.
6. Press the stop button to examine the frame collected.

Similarly, the entire frame from “SHUNYA to NAU” has been collected by repeating the abovementioned steps. Figures 8–10 show the spectrum of the spoken digits for different variations.

## 5. Proposed Model and Results

Suppose “S” is the target person's speech represented by *S*={*s*_1_, *s*_2_,…, *s*_*T*_} and “V” is the unobservable part of the speech dependent represented by *V*={*v*_1_, *v*_2_,…, *v*_*T*_}, then for statistically independent S and V, probability *P*(*x*_*t*_, *j*, *k*) can be calculated as follows:

(1) $$\begin{array}{c} P\left(x_{t},j,k\right)\int_{\infty }^{\infty }M\left(S;\sum_{s,j},\mu_{s,j}\right)M\left(x_{t}-S;\sum_{v,k},\;\mu_{v,k}\right), \end{array}$$

where ∑_*s*,*j*_ and ∑_*v*,*k*_ are weight covariance matrix and *μ*_*s*,*j*_ and *μ*_*v*,*k*_ are mean vectors, and *M* denotes the Gaussian density matrix.

Speaker-specific model *λ*_*s*_ in the maximum likelihood is given by

(2) $$\begin{array}{c} \lambda_{s}^{*}=\underset{\arg}{\max}P\left(XΙ\lambda_{x},\lambda_{v}\right),\\ =\underset{\arg}{\max}\prod_{j=1}^{J}\prod_{k=1}^{K}\prod_{t=1}^{T}w_{z,j}w_{z,k}P\left(x_{t}Ιj,k\right). \end{array}$$

So, given *λ*_*v*_ in (2) can be solved using the expectation maximization algorithm, starts with the initial model *λ*_*s*_ and estimate new one *λ*_*s*_^Ι^. The proposed model for verification is shown in Figure 7.

RETRACTED

Here, *P* (*X*Ι*λ*_*v*_, *λ*_*s*_^Ι^) ≥ *P*(*X*Ι*λ*_*v*_, *λ*_*s*_), and when testing is found to be unknown speech, then the system determines whether or not it is produced by the claimed speakers using the following equation:

(3) $$\begin{array}{c} \log\;P\left(YΙ\lambda_{v},\lambda_{s}\right)-\log\left(YΙ\lambda_{v}\right). \end{array}$$

It is satisfied when it is less than *θ*, and unsatisfied when greater than or equal to *θ*. Here, *Y* is the utterance cestrum feature and *θ* is the threshold level.

The efficiency of different coding techniques is shown in Table 4 represented graphically in Figure 11, where LPC means linear predictive coding, MFCC means Mel-frequency cepstral coefficient, and LPCC means linear prediction cepstral coefficient.

The linear predictive coding (LPC) is a technique for compressing the frequency spectrum of a digitized voice signal utilizing data from a linearly statistical model. It is broadly applied in auditory signal processing and speech analysis. The LPCC is based on linear prediction that provides the people articulatory system.

Moreover, the variation in the frequency spectrum is shown in Figures 12 and 13.

## 6. Conclusion

Using this speech-dependent health monitoring and management system, speech data can be collected from remote locations and can be accessed. As per the study, it is found that COVID-19 virus first affects our throat, and then it enters into the pumping area (heart). Therefore, in such a condition, a sample in the form of voice is collected from particular areas where COVID-19 patient is large in number and can be analyzed using such a model which helps to first detect his voice quality and matched with the original voice as saved in database. The proposed model provides a better management system without touching and maintains appropriate distance information that can be collected and processed for medical treatment. The future scope of this research is that it will reduce the chances to come into contact with a viral effected people in future. Any feature extraction approach can be imposed on that proposed model whose efficiency is found to be better to sample and analyze the speech signal to achieve good authentication. As per our analysis, MFCC found a good efficiency rate, i.e., 93.43% for the spoken digit, which may suit for further analysis. Blood sampling can be avoided using this method, and of course social distancing can also be maintained by remotely accessing the voice sample and proven to be a much better option for the society. Smart solution for the upcoming generation is required in terms of better facility, less pain, economical, and fast results. Therefore, such health care and management system is proved beneficial, and its implementation changes the face of health units in rural as well as urban areas.

RETRACTED

## Figures and Tables

**Figure 1:** Training in a speaker recognition system.

**Figure 2:** Speaker recognition testing system.

**Figure 3:** Principle shape of a closed set recognition system.

**Figure 4:** Principle structure of an addresser recognition system.

**Figure 5:** Gaussian mixture model with its feature space and corresponding 2-dimension.

**Figure 6:** Model for monitoring and management (assembled with the proposed model, Figure 7).

**Figure 7:** Proposed model for verification and authentication.

**Figure 8:** Spectrum of spoken digits.

**Figure 9:** Sampling of spoken digits.

**Figure 10:** Spectrum selection for complete spoken digits.

**Figure 11:** Efficiency of “SHUNYA” and “EK.”

**Figure 12:** Variation in the frequency spectrum of spoken digit “SHUNYA.”

**Figure 13:** Variation in frequency spectrum of spoken digit “EK.”

**Table 1:** Text-attached and self-reliant text process.

Verification of text-dependent	Verification using speech recognition	Verification with text-prompted	Verification with text-independent
Phase 1: S1: Using touch-tone keypad kindly enter your account number Caller1: 1234*∗*# Step2: S1: Please say your password Caller1: INDIAN S1: Thanks!	S1: Please say your account number. Caller1: 1234*∗*# S1: Thank you!	Phase 1: S1: Using touch-tone keypad kindly enter your account number Caller1:1234*∗*# Step 2: Computer please repeat 43–69 Caller: 43–69 S1: Kindly repeat 82–24 Caller1: 82–24 S1: Thanks!	Call centre ID: How can I help you Mr. Shrikant? Caller1: I want to transfer the amount 10,123 from my savings account with you to my foreign account in Nepal that I have opened. Agent: Please hold while I am fetching the information and have a look at that. Wait for a while, the computer is matching the identity of calling agent. Agent: Thanks! Process request

**Table 2:** Database of 50 speakers.

SL. No.	Name
0	Ambika_25F
1	Aditi_28F
2	Anil_24M
3	Anju_23F
4	Ankitraj_24M
5	Chandu_26M
6	Choti_18F
7	Deepak_26M
8	Deepmala_23F
9	Devmal_24M
10	Gauri_22F
11	Gopal_24M
12	Goutmi_23F
13	Hitan_24M
14	Isha_18F
15	Indira_24F
16	Kamal_25M
17	Kaushal_25M
18	Kiraan_18F
19	Lovley_26F
20	Mantu_24M
21	Navin_26M
22	Neetu_25F
23	Nitika_24F
24	Pankaj_27M
25	Parvathi_22F
26	Puja_24F
27	Prarthana_19F
28	Ramol_24F
29	Ravikant_24M
30	Ribha_21F
31	Sakshi_24F
32	Sanhita_23F
33	Sanjay_24M
34	Satyas_25M
35	Shaleen_23F
36	Shallu_23F
37	Shantanu_23M
38	Shipra_26F
39	Shital_24M
40	Sourav_25M
41	Sujjal_22M
42	Swati_23F
43	Sweta_22F
44	Toral_25F
45	Usharani_26F
46	Uttkal_25M
47	Vandana_19F
48	Vibha_19F
49	Vikash_26M

RETRACTED

**Table 3:** Parameters used for collecting data.

Parameters	Values
Total number of speakers	50
Single channel	16 KHz
Sampling rate	16 bit (for less quantization error)
Language	Hindi (phonetics is rich)
Repetition rate of each speaker	10 digits/minute

**Table 4:** Efficiency rate in % of individual feature extraction.

Hindi dialects	LPC (%)	MFCC (%)	LPCC (%)
0 (SHUNYA)	89.99	91.99	90.89
1_EK	88.12	92.23	89.98
2_DO	90.10	89.97	88.27
3_TEEN	87.26	89.25	88.12
4_CHAR	90.12	91.25	90.22
5_PANCH	92.29	90.23	91.67
6_CHEH	90.54	93.44	92.81
7_SAAT	89.11	90.23	92.64
8_AATH	90.78	94.10	90.21
9_NAU	91.34	93.43	87.66

## Data Availability

The data are used to support this study are available on request.
